The article "The Drosha-Independent MicroRNA6778-5p/GSK3β Axis Mediates the Proliferation of Gastric Cancer Cells" was published in 2022. Journal: Comput Intell Neurosci.

# The Drosha-Independent MicroRNA6778-5p/GSK3*β* Axis Mediates the Proliferation of Gastric Cancer Cells

**DOI:** 10.1155/2022/5932512

**Published:** 2022-09-30

**Authors:** Mingjun Ren, Li Xing, Wanping Wang, Wanying Bi, Wanjun Wu, Gui Jiang, Weiji Wang, Xingdong Liang, Manran Liu, Shifu Tang

**Affiliations:** ^1^Department of Laboratory Medicine, Liuzhou People's Hospital, Liu Zhou 545006, China; ^2^Liuzhou Key Laboratory of Precision Medicine for Viral Diseases, Liu Zhou 545006, China; ^3^Graduate School, Guangxi University of Chinese Medicine, Nanning 530000, China; ^4^Department of Laboratory Medicine, Liuzhou Traditional Chinese Medicine Hospital, Liu Zhou 545006, China; ^5^Gastrointestinal Surgery, Liuzhou People's Hospital, Liu Zhou 545006, China; ^6^Laboratory Medical College, Chongqing Medical University, Chongqing 400016, China

## Abstract

**Background:**

Gastric cancer (GC) is a primary cause of cancer death around the world. Previous studies have found that Drosha plays a significant role in the development of tumor cells. Soon after, we unexpectedly found that the expression of microRNA6778-5p (miR6778-5p) is unconventionally high in the gastric cancer cells low-expressing Drosha. So, we designed the Drosha interference sequence and recombined it into a lentiviral vector to construct Drosha knockdown lentivirus and transfected the Drosha knockdown lentivirus into gastric cancer cells to establish Drosha knockdown gastric cancer cell lines. We aimed to explore the effect of microRNA6778-5p on the proliferation of gastric cancer cells with Drosha knockdown and its intrinsic mechanism.

**Methods:**

We designed the Drosha interference sequence and recombined it into a lentiviral vector to construct Drosha knockdown lentivirus and transfected the Drosha knockdown lentivirus into gastric cancer cells to establish Drosha knockdown gastric cancer cell lines. After transfecting miR6778-5p mimics and inhibitor into gastric cancer cell lines with Drosha knockdown, the expression levels of miR6778-5p mimics in Drosha low-expressing gastric cancer cells increased, while miR6778-5p inhibitor decreased the expression levels of miR6778-5p. The Cell Counting Kit-8 (CCK-8) experiment was used to detect the proliferation ability of gastric cancer cells after overexpression or knockdown of miR6778-5p and bioinformatics predicted the relationship between miR6778-5p and glycogen synthase kinase-3*β* (GSK3*β*).

**Results:**

After infection with the Drosha knockdown lentivirus, Drosha's mRNA and protein levels were significantly downregulated in gastric cancer cells. The expression levels of miR6778-5p mimics in Drosha low-expressing gastric cancer cells increased, while miR6778-5p inhibitor decreased the expression levels of miR6778-5p. Overexpression of miR6778-5p significantly enhanced the proliferation ability of Drosha low-expression gastric cancer cells; on the contrary, knocking down miR6778-5p weakened the proliferation ability of Drosha low-expression gastric cancer cells. Bioinformatics predicted that miR6778-5p targeted glycogen synthase kinase-3*β* (GSK3*β*) and the mRNA and protein levels of GSK3*β* decreased significantly after overexpression of miR6778-5p.

The article "The Drosha-Independent MicroRNA6778-5p/GSK3β Axis Mediates the Proliferation of Gastric Cancer Cells" was published in 2022. Journal: Comput Intell Neurosci.

**Conclusion:**

miR6778-5p promotes the proliferation of Drosha low-expressing gastric cancer cells by targeting GSK3*β*.

## 1. Introduction

Gastric cancer is a malignant tumor with high morbidity and mortality worldwide [1]. There are approximately 110000 new cases and 770000 deaths annually, accounting for 5.6% in total number of cancers and 7.7% in total number of cancer deaths [2]. Although some progress has been made in clinical therapy, the long-term survival for patients with advanced cancer remains poor, with a five-year survival rate of only 12% [3]. Among them, the recurrence of GC is a principal element affecting the survival rate of advanced patients. So, it is urgent to explore the underlying molecular mechanism of the development process of GC and is beneficial to discover new therapy targets of gastric cancer.

Drosha belongs to the endoribonuclease III superfamily. As a core nuclease, Drosha performs the initial step of miRNA processing by cutting the hairpin structure embedded in the primary transcript in the nucleus [4]. Drosha is significant for microRNA processing, which can convert the initial microRNA (pri-miRNA) into the precursor microRNA (pre-miRNA) in the nucleus, laying foundation for the maturation of microRNA [5]. Drosha's RNA interference leads to massive accumulation of pri-miRNA in vivo, with consequent reduction in pre-miRNA and mature miRNA. In addition, there is also a mirtron pathway that does not rely on Drosha to cause miRNA biogenesis, which can suppress or promote cancer [6, 7]. Indeed, previous research has found that Drosha plays an extremely vital part in tumor cell development, and the abnormal expression of Drosha will lead to changes in the expression of microRNA [8, 9]. Especially in some Drosha knockout models, some miRNA expressions are upregulated instead [10]. As we all know, microRNAs are a class of highly conserved and short-stranded non-coding RNAs that partake in the regulation of cell multiplication, apoptosis, and metabolism, and their abnormal expression also affects the progression of tumors [11–13]. The currently recognized mechanism of microRNA's influence on tumors is through targeted inhibition of its related genes to perform their functions [14, 15]. Our preliminary research found that Drosha knockdown in GC cells reduces the migration of cancer cells, accompanied by upregulation or downregulation of miRNA, which is a poor prognostic factor. Of note, we unexpectedly found that microRNA6778-5p (miR6778-5p) expression is unconventionally high in the gastric cancer cells low-expressing Drosha, while miR6778-5p is a non-canonical miRNA type that does not depend on Drosha, spliced from the SHMT1 intron [16]. To clarify the molecular mechanism of miR6778-5p regulating the low expression of Drosha in gastric cancer, we used the miRTarBase and TargetScan databases to find that GSK3*β* was a potential target gene of miR6778-5p. c-Myc, a class of target genes, is upregulated to accelerate cell multiplication by *β*-catenin. Meanwhile, GSK3*β* takes a pivotal effect on controlling cell proliferation by negatively regulating the transcription activity of *β*-catenin [17]. To our knowledge, till now miR6778-5p/GSK3*β* axis has no relevant reports on cell multiplication. It is unclear that whether miR6778-5p has an essential part via GSK3*β* in accelerating GC cell multiplication with Drosha knockdown.

The article "The Drosha-Independent MicroRNA6778-5p/GSK3β Axis Mediates the Proliferation of Gastric Cancer Cells" was published in 2022. Journal: Comput Intell Neurosci.

In this study, we found that mir-6778-5p played a positive role in GC cell proliferation. The upregulation of miR6778-5p results from Drosha interference in GC cells. The mimics and inhibitors of miR6778-5p can enhance or inhibit the multiplication of GC cells low-expressing Drosha. Moreover, miR6778-5p regulates the multiplication behavior of GC cells low-expressing Drosha by targeting GSK3*β*. In short, the microRNA6778-5p/GSK3*β* axis mediates the multiplication of GC cell lines low-expressing Drosha.

## 2. Methods

### 2.1. Cell Lines and Culture Conditions

The GC cell lines MGC-803 and SGC-7901 needed for the experiment were presented by Professor Yang Ke from Beijing Cancer Institute (Beijing, China). These cells were incubated in RPMI1640 (Gibco, USA) or DMEM (Gibco, USA) supplemented with 10% FBS (Gibco, USA). Cells were cultured in humidified air at 37°C containing 5% CO2.

### 2.2. Transfection Assay

The cells were placed in 2 ml whole culture medium with 1 × 10^5^ cells per well in in 6-well plates, respectively. Infected cells with the lentivirus contain Drosha-shRNA sequence (5′-AACGAGUAGGCUUCGUGACUU-3′) or negative control sequence (5′-UUCUCCGAACGUGUCACGUTT-3′) (GenePharma Co., Ltd. Shanghai) when the cell density reached 60%. Furthermore, they were screened with 1 *μ*g/ml puromycin, establishing MGC-803/Drosha KD or SGC-7901/Drosha KD cell lines, respectively. Similarly, when reaching 60% confluence in 6-well plates, cells were treated with 100 pmol miR6778-5p mimics, 100 pmol miR6778-5p inhibitor, or the corresponding random sequence RNA Oligo (negative control) (GenePharma Co., Ltd. Shanghai) separately according to the protocol of Lipofectamine 2000 transfection kit (Invitrogen, USA).

The article "The Drosha-Independent MicroRNA6778-5p/GSK3β Axis Mediates the Proliferation of Gastric Cancer Cells" was published in 2022. Journal: Comput Intell Neurosci.

### 2.3. RNA Extraction and qRT-PCR Detection

Total RNA was isolated from the corresponding gastric cancer cells using Trizol (Invitrogen, USA). RNA quantity was detected by spectrophotometry and by agarose gel electrophoresis. qRT-PCR was done using the PrimeScript RT reagent kit and SYBR Premix Ex TaqTM (Takara, Japan) following the manufacturer's instruction. Two-step amplification, Holding stage: 95°C, 30 s (1 cycle); Cycling stage: 95°C, 5 s–60°C, 34 s (40 cycles); Melt curve stage: 95°C, 15 s–60°C, 60 s–95°C, 15 s (1 cycle). *β*-Actin was used as the internal control and primer sequences were: Drosha: 5′-CGATGATGCAGGGAAACACATG-3′ (forward) and 5′-TTATTTCTTGATGTCTTCAGTCT-3′ (reverse). miR6778-5p: 5′-GCGAGTGGGAGGACAGGAG-3′ (forward) and 5′-ATCCAGTGCAGGGTCCGAGG-3′ (reverse). GSK3*β*: 5′-CCTTAACCTGCTGCTGGACT-3′ (forward) and 5′-AGCTCTGGTGCCCTGCCAGAT-3′ (reverse). *β*-Actin: 5′-AGGGGCCGGACTCGTCATACT-3′ (forward) and 5'-GGCGGCACCACCATGTACCCT-3′ (reverse).

### 2.4. Western Blot

Western blot assays were done as described previously [18]. Cells were harvested with RIPA buffer (Beyotime, China) to extract total protein measured with the BCA protein assay kit (Beyotime, China), isolated by 10% SDS-PAGE gel electrophoresis. The protein is transferred to the PVDF membrane. After incubating with primary antibodies overnight at 4°C, the corresponding HRP-conjugated secondary antibodies (Beyotime, China) were subsequently applied and immunodetection was performed using the enhanced chemiluminescence system (Cool-Imager).

### 2.5. Cell Multiplication Assay

The cell multiplication rate was detected by the CCK-8 assay (Beyotime, China). Cells were placed on 96-well plates with 3 × 103 cells per well. Cells were processed by 100 pmol miR6778-5p mimics and 100 pmol miR6778-5p inhibitor (GenePharma Co., Ltd., Shanghai) at different points in time when 60% confluence was reached. After the treatment, the medium was discarded. A small orifice was placed at 10 μL CCK-8 reagent and continued to incubate for 4 hours before adding DMSO (200 μl per well), and shaken slowly on a shaker for 10 min. Measurement was performed by using an absorbance meter.

### 2.6. Statistical Analysis

Statistical analysis was performed using the SPSS standard version 19.0 software. The data were presented as mean ± standard deviation $\left(\bar{x}\pm s\right)$. Each experiment was repeated at least 3 times. Pairwise comparisons between groups were performed using the LSD *t*-test, and P < 0.05 was considered statistically significant.

The article "The Drosha-Independent MicroRNA6778-5p/GSK3β Axis Mediates the Proliferation of Gastric Cancer Cells" was published in 2022. Journal: Comput Intell Neurosci.

## 3. Results

### 3.1. The Expression of miR6778-5p Increases in GC Cells with Drosha Knockdown

To investigate the role of miR6778-5p in GC low-expressing Drosha, we constructed a vector lentivirus with the Drosha interference sequence and then infected MGC-803 GC cell and SGC-7901 GC cell with the virus to establish GC cell lines with Drosha low expression. The mRNA and protein expression of Drosha were significantly reduced compared with the control group (Figures 1(a) and 1(b)) and the miR6778-5p expression was visibly increased (Figure 1(c)) in MGC-803 and SGC-7901 cells transfected with the Drosha knockdown lentivirus.

### 3.2. Overexpression of miR6778-5p Promotes the Multiplication of GC Cells Low-Expressing Drosha

To demonstrate whether miR6778-5p regulates the multiplication of GC cells low-expressing Drosha, we transfected Drosha low-expressing GC cells (MGC-803/Drosha KD and SGC-7901/Drosha KD) with miR6778-5p mimics and evaluated the proliferation potential change of MGC-803/Drosha KD and SGC-7901/Drosha KD treated with miR6778-5p mimics. As shown in Figures 2(a) and 2(b), the expression levels of miR6778-5p increased significantly and enhanced the proliferation ability of MGC-803/Drosha KD and SGC-7901/Drosha KD cells treated with miR6778-5p mimics. These results showed that miR6778-5p has a positive influence on multiplication of GC cells low-expressing Drosha.

### 3.3. Knockdown of miR6778-5p Inhibits the Multiplication of Low-Expression Drosha GC Cells

In order to further verify whether miR6778-5p controls the proliferation ability of Drosha low-expressing GC cells, we transferred the inhibitor of miR6778-5p to lower expression Drosha GC cells and then evaluated the proliferation potential change of MGC-803/Drosha KD and SGC-7901/Drosha KD treated with miR6778-5p inhibitor. Expectedly, the expression levels of miR6778-5p decreased and the proliferation ability reduced significantly in MGC-803/Drosha KD and SGC-7901/Drosha KD cell lines after treating with miR6778-5p inhibitor (Figures 3(a) and 3(b)). It is confirmed once again that miR6778-5p promotes the multiplication capacity of GC cells low-expressing Drosha.

### 3.4. The miR6778-5p/GSK3*β* Axis Mediates the Multiplication Potential of Drosha Low-Expressing GC Cells

As is well-known, microRNA regulates human tumor development by binding to the 3′UTR end of its target genes to inhibit the expression of coding target genes. We searched the microRNA target gene databases to find that GSK3*β* was a potential target gene of miR6778-5p (Figure 4(a)). In order to investigate the intrinsic molecular mechanism of miR6778-5p regulating the multiplication potential of GC cells, we conducted experiments to demonstrate the effect of miR6778-5p on the expression levels of GSK3*β*, a key negative regulator of cell cycle. According to the experimental results, we observed that after overexpressing miR6778-5p in Drosha low-expressing GC cells, the mRNA and protein expression of GSK3*β* decreased obviously (Figure 4(b)). On the contrary, after knocking down miR6778-5p in Drosha low-expressing GC cells, the mRNA and protein expression of GSK3*β* increased apparently (Figure 4(c)). The above results showed that the miR6778-5p/GSK3*β* axis plays an important role in promoting the proliferation of gastric cancer cells low-expressing Drosha.

The article "The Drosha-Independent MicroRNA6778-5p/GSK3β Axis Mediates the Proliferation of Gastric Cancer Cells" was published in 2022. Journal: Comput Intell Neurosci.

## 4. Discussion

The intrinsic mechanism of gastric cancer carcinogenesis is not fully clarified. Abnormal proliferation, one of the cancer hallmarks, is the chief death cause of gastric cancer patient. Although there is great progress in gastric cancer treatment including radiotherapy, neoadjuvant chemotherapy, molecular targeted therapy, and immunotherapy, gastric cancer, especially advanced gastric cancer, is hard to cure [19]. Therefore, there is an urgent need to reveal the mysterious nature of gastric cancer for finding new treatment targets of GC. In our previous research, we discovered that after Drosha knockdown, the biological behavior of gastric cancer cells will be changed [20]. In this study, Drosha-independent miR6778-5p was found to promote the multiplication of GC cells with Drosha knockdown via inhibiting the expression of its target gene GSK3*β*. To the best of our knowledge, it is firstly reported that the Drosha-independent miR6778-5p/GSK3*β* axis mediates the multiplication of GC cells low-expressing Drosha.

miR6778-5p biogenesis increases in gastric cancer cells with Drosha knockdown. Pri-miRNAs are the primary transcripts which evolve into mature miRNAs after two splicing [21]. Drosha, an endonuclease RNase III enzyme, is necessary for cleaving the primary transcripts of miRNAs, the first step of microRNA maturation process [21]. Besides, Drosha aberrant expression plays a vital part in the pathological process of cancer. Although it is controversial whether Drosha promotes or suppresses the pathological process of cancer [22], Drosha behaves as an oncogene in gastric cancer [16, 20]. Drosha knockdown expectedly reduces the expression of many miRNAs but increases the expression of many other miRNAs [20], indicating that the biogenesis of the upregulated miRNAs is Drosha-independent. This miRNA, obtained by direct splicing through introns and bypassing Drosha, is also called the mirtron pathway [23]. Indeed, the biogenesis of miR-6778-5p is non-canonical in GC cells with Drosha knockdown [16]. However, the non-canonical mechanism of miR-6778-5p biogenesis remains to be clarified in GC cells with Drosha knockdown.

miR-6778-5p has an active effect upon the multiplication of GC cells with Drosha knockdown via targeting GSK3*β*. Drosha silence impedes the invasion of GC cells but does not affect other malignant behaviors such as proliferation [16, 20], suggesting that miR-6778-5p could regulate the multiplication of low-expressing Drosha GC cells. MicroRNA is a type of non-coding RNA, which regulates gene expression at the post-transcriptional level by targeting mRNA degradation and/or inhibiting its translation, thereby regulating the development of cancers [24]. It is predicted that GSK3*β* is a potential target gene of miR6778-5p through searching the microRNA target gene databases (Figure 4(a)). GSK3*β* is a multifunctional serine/threonine kinase. Now it has been proved that GSK3*β* acts as a negative regulator in Wnt/*β*-catenin, PI3K/AKT, and other signaling pathways [25–27]. Upregulation of miRNA-29a can reduce GSK3*β* protein expression in colorectal cancer cells and inhibit Wnt/*β*-catenin signaling pathway [28]. In this research, we demonstrated that miR6778-5p inhibits the expression of GSK3*β* via binding the 3′UTR of GSK3*β* mRNA in gastric cancer cells with Drosha knockdown. As far as we know, it was firstly found that the miR-6778-5p/GSK3*β* axis promotes the cell proliferation.

The article "The Drosha-Independent MicroRNA6778-5p/GSK3β Axis Mediates the Proliferation of Gastric Cancer Cells" was published in 2022. Journal: Comput Intell Neurosci.

Circular RNAs (circRNAs) are considered a neoteric type of non-coding RNA with organization, structure, time, and space specificity characterized by a covalently closed-loop structure involved in modulating gene expression by regulation of miRNA function, transcription, and protein [29]. Growing study showed that circRNAs contribute to many physiological and pathological processes, including the pathological progression of cancer [30]. CircRNAs perform their biological functions mainly via the circRNA-miRNA-mRNA regulatory network [18, 31, 32]. It remains to be explored whether Drosha-independent miR6778-5p exerts positive effect on the multiplication of GC cells through the circRNA-miRNA-mRNA regulatory network.

## 5. Conclusions

In a nutshell, this research proves that the Drosha-independent microRNA6778-5p/GSK3*β* axis mediates the multiplication of GC cells. These discoveries will provide in-depth knowledge of the mechanisms by which Drosha-independent miRNAs promote the abnormal multiplication of GC cells and original therapeutic markers of gastric carcinoma.

## Figures and Tables

**Figure 1:** Drosha-independent miR6778-5p expression increases in gastric cancer cells. (a) The mRNA expression levels of Drosha were determined by qRT-PCR in gastric cell lines with Drosha knockdown (^*∗∗*^*P* < 0.05). (b) The protein expression levels of Drosha were verified by WB in gastric cell lines with Drosha knockdown (^*∗∗*^*P* < 0.05). (c) The expression levels of miR6778-5p were detected by qRT-PCR in gastric cancer cells low-expressing Drosha (^*∗∗*^*P* < 0.05).

The article "The Drosha-Independent MicroRNA6778-5p/GSK3β Axis Mediates the Proliferation of Gastric Cancer Cells" was published in 2022. Journal: Comput Intell Neurosci.

**Figure 2:** Overexpression of miR6778-5p promotes the proliferation of gastric cancer cells with Drosha knockdown. (a) The expression levels of miR6778-5p were evaluated by qRT-PCR (^∗∗^P<0.05). (b) Growth curves were observed using the CCK8 assay (^*∗∗*^*P* < 0.05).

**Figure 3:** miR6778-5p silence inhibits the proliferation of gastric cancer cells with Drosha knockdown. (a) The expression levels of miR6778-5p were evaluated by qRT-PCR (^*∗∗*^P<0.05). (b) Growth curves were observed using the CCK8 assay (^*∗∗*^P<0.05).

**Figure 4:** The miR6778-5p/GSK3*β* axis mediates the proliferation of Drosha low-expressing gastric cancer cells. (a) miR6778-5p acts on the 275–281 sites in the UTR of GSK3*β* mRNA through its seed sequence. (b) The mRNA and protein expression levels of GSK3*β* were detected by qRT-PCR or WB in MGC-803/Drosha KD or SGC-7901/Drosha KD cell lines after being transfected with miR6778-5p mimics (^*∗∗*^*P* < 0.05). Immunoblotting analyses were performed with the indicated antibodies. (c) The mRNA and protein expression levels of GSK3*β* were determined by qRT-PCR or WB in MGC-803/Drosha KD or SGC-7901/Drosha KD cell lines after being transfected with miR6778-5p inhibitor (^*∗∗*^*P* < 0.05). Immunoblotting analyses were performed with the indicated antibodies.

## Data Availability

The data used in this study are available from the corresponding author upon request.
